The article "Dynamic Analysis of College Physical Education Teaching Quality Evaluation Based on Network under the Big Data" was retracted in 2023. Reasons: unreliable results or conclusions; concerns about the data; concerns about the results or conclusions; concerns about the peer review.

# Dynamic Analysis of College Physical Education Teaching Quality Evaluation Based on Network under the Big Data

**DOI:** 10.1155/2021/5949167

**Published:** 2021-12-23

**Authors:** Bin Feng

**Affiliations:** Zhixing College, Hubei University, Wuhan 430000, Hubei, China

## Abstract

Improving the quality of college physical education is of great significance to facilitating the integrated development of students' psyches and physical. Establishing a more systematic, effective, and social training needs of education quality evaluation hierarchy is also the centerpiece of the college physical culture education administration. Massive information technology provides new conception and methods to this, and supply advantage sustains for furtherance the education ecology development. Based on the network education system, this paper uses big data to quantify the evaluation indexes of physical education teaching, so as to actualize the timely dynamic evaluation of the process that is physical teaching and learning. This essay constructs the evaluation index system of college physical education teaching quality by combining mensurable and qualitative methods. On the basis of previous studies, an evaluation model of college physical education teaching quality based on artificial intelligence mass data calculation is designed. The experiment authenticates that the model evaluation risk coefficient is 1.93 lower than the optimized model. The experiment also proves that the model is conducive to elevating the education quality.

## 1. Introduction

### 1.1. Background

With the rapid development of education, China attaches more importance to physical education. In college physical education, teaching quality is a significant relationship to students' basic physique, students' all-round growth, and the future of the motherland. There are many shackles still exist in the physical education evaluation sequence in college step, such as paying too much attention to qualitative evaluation and result evaluation, taking achievements as reference, teaching practice not included in the evaluation system, and lack of effective incentive measures for teachers. How to adopt positive and valid functions to improve the current educational performance assess quota hierarchy and scientifically and reasonably evaluate the quality of physical education in colleges and universities is a problem worthy of our in-depth study.

In the meantime, with the ceaseless integration of information and communication technology into our lives, the environment of education has changed, and online education has exploded. Web education has a great effect in university study process. Moreover, increasing higher education institutions now have their own Web education system for teaching management [1]. In the past, due to the limitation of objective conditions, the evaluation of physical education teaching quality in colleges and universities is usually intermittent and result-oriented, and cannot accurately reflect the quality of teaching process.

Under the tide of big data era, we can obtain intuitive data massage in the teaching process with the help of massive data, so as to optimize teaching and improve the quality of education and teaching. Therefore, it is urgent to consider how to optimize the education quality evaluation system and dynamically evaluate the curriculum quality by computing with big data, which is also what this paper intends to discuss.

### 1.2. Significance

College physical education based on network is a complex project of multi-factor system optimization, which not only needs theoretical teaching optimization, but also needs students' real-time feedback supervision optimization, which is more interactive than other disciplines. As a result, it has become a realistic need for the comprehensive informational transformation of educational evaluation methods. Therefore, the significance of dynamic evaluation of physical education quality by computing with big data and computer technology has become clear [2]. This paper studies this from the theoretical and empirical perspective, in order to obtain highly differentiated evaluation data under deep learning, construct a more scientific evaluation index system, and promote the quality and efficiency of college physical education under the information environment.

### 1.3. Related Work

Teaching quality evaluation is an important way of school quality management and an important means to promote the pace of education. With the deepening of the concept of “life education,” the quality of physical education has attracted attention from all walks of life. With the development of a large amount of data technology, more and more people have begun to study the concept of big data for evaluating the quality of physical education teaching.

Based on the analysis of the effect of physical education in colleges and departments, Wang adopted the fuzzy evaluation method, including students' awareness of participating in physical education, students' individual expend, students' lifelong physical education, students' physical education ethics, and team spirit. According to the teaching achievement evaluation index system, the fuzzy comprehensive evaluation of physical education teaching quality is obtained. At the same time, the optimization suggestions for the evaluation model are put forward [3]. But it has not applied the optimized evaluation model in practice. Applying *w* obtains three principal components of input and three principal components of output. Based on the principle of index construction, the above results are obtained by using principal component analysis to eliminate the correlation between indexes. In addition, a data envelopment analysis model was established to compare the school-running efficiency of these 24 universities and understand the school-running efficiency and difference of each university [4]. However, his research content is a little general and did not put forward specific suggestions for the problems of running colleges and universities. Zhao analyzed and studied the status quo of physical education teaching quality evaluation system in colleges and universities through the method of logical analysis and proposed the corresponding design strategy of evaluation system of physical education teaching quality based on the characteristics of social development at the present stage [5]. The evaluation subject in the evaluation system is too single and does not start from multilevel. Huang put forward the problems existing in traditional physical education teaching from multiple angles and put forward the results-oriented reform measures in college physical education teaching from the aspects of rational development of training plans and construction of three-level physical education [6]. Results-oriented teaching reform is easy to be one-size-fits-all without scientific integration of process-based evaluation system. Williams screened a random sample of 56 institutions to determine whether they offered PE and CPE courses. The results show that more than 70% of institutions require physical education as a general education requirement or offer CPE. Further studies show that many dependent variables of course content analysis standards, including course composition, description and objectives, curriculum, and evaluation, all score at 50% or higher [7]. The results show that physical education is increasingly valued, but the study does not suggest an improved evaluation system. Based on the theory of multiple intelligences, Zhao based on the analytic hierarchy process; according to the weight of each evaluation index and the participation degree of fuzzy evaluation information, this paper puts forward the fuzzy comprehensive evaluation model of college physical education and constructs the evaluation index system and management steps of physical education teaching from three aspects of teaching, and teaching and learning [8]. This model is an attempt to evaluate PE teaching effectively and has been proved in the experiment. Sun not only made a theoretical discussion on the effectiveness of physical education teaching quality, but also made an empirical analysis on the existing physical education teaching quality by using the evaluation model. The results of experimental analysis show that most students hold a positive attitude toward the effectiveness of physical education teaching quality defined in the evaluation [9]. Sun research provides support for universities to improve teaching quality, but there is no experimental application to verify the effectiveness of teacher evaluation model. Li used analytic hierarchy process to evaluate and improve college physical education, in order to improve the efficiency of interactive physical education. He put forward the problems faced in the process of network teaching and used the network teaching system to realize the real-time interaction and evaluation process [10]. The whole functional block model he mentioned is still inadequate in evaluating functional diversity.

### 1.4. Innovation Point

The professional application of advanced data advances educational management. This paper is supported by deep mining of big data. The innovation of this article has the following three points: (1) multiple quantitative analysis methods are tried to determine the weight allocation of indicators and their validity is checked and compared; (2) try to construct a scientific and dynamic college physical education evaluation system and method based on network framework; and (3) it breaks through the traditional evaluation method of school teaching quality, which is conducive to promoting the informational and data of education management.

## 2. Evaluation Mean of College Physical Education Standard on account of the Massive Data

### 2.1. Massive Data Technology and Continuous Data Acquisition Method

Relying on cloud computing, big data mining technology can carry out distributed information mining for massive data and process meaningful data [11]. It is an irresistible trend to apply massive data calculate to educational analysis and management. The data obtained by big data are far more objective and real than traditional data collection methods such as questionnaires and artificial judgments, because the objects of data collected can be ignorant and will not worry about human relationships [12]. The processing of massive information is more accurate, with more dimensions and full dynamic process. It can avoid the disadvantages of the previous education decision-making, and it is a brand new attempt and a leap in quality for education management. Big data technology is inseparable from storage technology, perception technology, and cloud computing, which constitute the whole process of data collection, processing, storage, and result formation [13, 14]. The specific structure is shown in Figure 1.

Big data are a new field of machine learning. Its purpose is to study how to automatically extract multilevel feature representation from data. Its basic idea is to extract features from the original data through a series of nonlinear transformations from low to high, from concrete to abstract, and from general to concrete. Deep learning not only changes the traditional machine learning methods, but also affects human understanding of cognition [15]. At present, breakthroughs have been made in the fields of speech recognition, image understanding, natural language processing, and so on.

### 2.2. Education Quality Assessment Methods

According to different subjects, educational evaluation methods can be divided into student evaluation, peer evaluation and peer evaluation, teacher self-evaluation, education department evaluation, and evaluation of other evaluation agencies [16]. From the point of view of the whole link of education and teaching, it also includes formative evaluation, process evaluation, and termination evaluation. In terms of methods, it can be divided into two categories: qualitative evaluation and quantitative evaluation. Qualitative evaluation focuses on the subjective judgment of education quality based on the existing knowledge and experience. Quantitative evaluation is an analysis method based on data, fuzzy mathematics, and statistics [17].

Generally speaking, scientific evaluation methods should be comprehensive, combining qualitative and quantitative evaluation, formative and summative evaluation, and evaluation of different subjects [18]. The research direction is teaching level evaluation supported by big data and basis of this paper, so quantitative analysis is particularly important, which can help us determine the weight of evaluation factors and related indicators through algorithms. The following focuses on the commonly used analysis method [19].

#### 2.2.1. Fuzzy Comprehensive Evaluation Method

Fuzzy comprehensive evaluation method is a kind of evaluation model, which can realize qualitative and quantitative evaluation. This method can combine deterministic factors and random factors for overall evaluation and is often used to determine teaching quality indicators and weights [20]. Assume that the evaluation index set composed of *M* factors is *S*={*s*_1_, *s*_2_,…*s*_*m*_}. On the basis of set *I*, set *P*={*p*_1_, *p*_2_,…*p*_*n*_}  is composed of *n* kinds of decisions. Since each factor has different influences on things, the weight distribution of factors needs to be determined, which is regarded as the fuzzy set of I and marked as

(1) $$\begin{array}{c} O=\left\{o_{1},o_{2},\ldots o_{m}\right\}\in F\left(I\right), \end{array}$$

where *o*_*i*_(*i*=1，2，3,…, *m*) represents the weight of the *i*th factor and *n* judgments are not absolutely yes or no. Therefore, comprehensive judgment should also be regarded as the fuzzy set on *p*, denoted as

(2) $$\begin{array}{c} R=\left\{r_{1},r_{2},\ldots r_{n}\right\}\in F\left(P\right), \end{array}$$

where *r*_*i*_(*i*=1，2，3,…, *n*) reflects the position of the ith judgment in the whole population [21].

Therefore, fuzzy evaluation has three basic factors: factor set *I*; evaluation set *p*; single factor evaluation, also known as fuzzy mapping;

(3) $$\begin{array}{c} f:s⟶F\left(P\right),\\ s_{i}\mapsto f:s=\left(b_{i1},b_{i2},\ldots ,b_{in}\right). \end{array}$$

Fuzzy relation can be induced by *f*

(4) $$\begin{array}{c} B=\left(\begin{array}{c} f\left(s_{1}\right)\\ f\left(s_{2}\right)\\ \ldots \\ f\left(s_{m}\right) \end{array}\right)=\left(\begin{array}{c} b_{11},b_{12},\ldots ,b_{1n}\\ b_{21},b_{22},\ldots ,b_{2n}\\ \ldots \\ b_{m1},b_{m2},\ldots ,b_{mn} \end{array}\right). \end{array}$$

*B* induces a fuzzy transformation

(5) $$\begin{array}{c} V_{B}:F\left(I\right)⟶F\left(P\right),\\ O\mapsto V_{B}\left(O\right)=O{}^{\circ}B. \end{array}$$

(*S*, *P*, *B*) constitutes a fuzzy comprehensive evaluation model, and input the weight distribution *O* into it to obtain a comprehensive evaluation

(6) $$\begin{array}{c} R=O{}^{\circ}B=\left\{r_{1},r_{2},\ldots r_{n}\right\},\\ \left\{r_{1},r_{2},\ldots r_{n}\right\}=\left\{o_{1},o_{2},\ldots o_{m}\right\}{}^{\circ}\left(\begin{array}{c} b_{11},b_{12},\ldots ,b_{1n}\\ b_{21},b_{22},\ldots ,b_{2n}\\ \ldots \\ b_{m1},b_{m2},\ldots ,b_{mn} \end{array}\right). \end{array}$$

After *R* is obtained, the membership function can be used to obtain the evaluation result.

#### 2.2.2. Gray Relational Analysis Method

Gray relational analysis method is proposed for the factors with neither empirical data nor uncertainty. This method quantifies the problems that are difficult to conduct qualitative. The correlation degree of all relevant elements in the system is measured by the correlation degree analysis method [22]. Assume that the reference sequence containing *α* is

(7) $$\begin{array}{c} Y_{0}=\left\{y_{01}，y_{02},\ldots ,y_{0\alpha }\right\}. \end{array}$$

Suppose there are *T* objects in the evaluation set. Then, the comparison sequence composed of *α* factor of the ith object is

(8) $$\begin{array}{c} Y_{i}=\left\{y_{i1}，y_{i2},\ldots ,y_{i\alpha }|\left(i=1，2,\ldots ,t\right)\right\}. \end{array}$$

Carry out dimensionless processing on the data, and then calculate the absolute value of the difference between the reference and comparison sequences at different points:

(9) $$\begin{array}{c} \Delta_{0i}\left(w\right)=\left|Y_{i}\left(w\right)-Y_{0}\left(w\right)\right|,\;\left(i=1,2,\ldots ,t;w=1,2,\ldots \alpha \right). \end{array}$$

Then, calculate the minimum difference and maximum difference within and between sequences:

(10) $$\begin{array}{c} \Delta_{\min}=\underset{i}{\min}\underset{j}{\min}\Delta_{0i}\left(w\right),\\ \Delta_{\text{man}}=\underset{i}{\max}\underset{j}{\max}\Delta_{0i}\left(w\right),\\ i=1,2,\ldots ,t;w=1,2,\ldots \alpha ；j=1,2,\ldots \alpha . \end{array}$$

The calculation formula of correlation coefficient in reference sequence and comparison sequence is as follows:

(11) $$\begin{array}{c} \sigma_{0i}=\frac{\Delta_{\min}+\theta \times \Delta_{\text{man}}}{\Delta_{0i}\left(w\right)+\theta \times \Delta_{\text{man}}}, \end{array}$$

where *θ* is the resolution coefficient greater than 0 and less than 1, and the smaller *θ* value is, the higher the resolution of the correlation degree [23].

Through the above calculation, the grey correlation sequence composed of *α* grey correlation coefficients of the ith object can be obtained as follows:

(12) $$\begin{array}{c} \sigma_{i}=\left(\sigma_{0i}\left(1\right),\sigma_{0i}\left(2\right),\ldots ,\sigma_{0i}\left(w\right)\right). \end{array}$$

Finally, the weighted processing method is used to calculate the correlation degree:

(13) $$\begin{array}{c} \varepsilon_{i}=\sum_{j=1}^{\alpha }\sigma_{i}\left(j\right)\cdot W\left(j\right),\;i=1,2,\ldots ,t;w=1,2,\ldots \alpha , \end{array}$$

where *ε*_*i*_ is the grey correlation degree value, *W*(*j*) is the weight of each parameter, and *W*(*j*) ≥ 0；∑_*j*=1_^*α*^*W*(*j*)=1.

#### 2.2.3. Analytic Hierarchy Process

Analytic hierarchy process (AHP) is used to calculate the weight coefficient of each factor in comprehensive evaluation. It is a systematic method combining quantitative and qualitative methods and is solved by matrix [24]. First of all, the teaching quality evaluation objectives should be decomposed layer by layer until they are subdivided into quantifiable factors. The weight calculation method of two-layer factor indicators is given as follows.

*A* matrix:

(14) $$\begin{array}{c} M=\left[\begin{array}{ccc} A_{11} & \cdots & A_{1\alpha }\\ \vdots & \ddots & \vdots \\ A\alpha 1 & \cdots & A_{\alpha \alpha } \end{array}\right],\\ M\gamma =\lambda_{\max}\cdot \gamma . \end{array}$$

The eigenvector corresponding to the maximum eigenvalues of *M* can be obtained by using the formula, and the weight distribution of each factor can be obtained by normalizing the eigenvector *γ.*

Whether the weight distribution obtained by the above calculation is reasonable and effective requires consistency test of the matrix. In formula (15), CI and RI are the general consistency index and average random consistency index of the matrix. CR is the stochastic uniformity ratio obtained from the ratio of the previous two. If CR < 0.10 or Δ_max_= *α*, CI=0, this matrix is acceptable. Otherwise, factors in the matrix need to be modified.

(15) $$\begin{array}{c} \text{CR}=\frac{\text{CI}}{\text{RI}}. \end{array}$$

#### 2.2.4. Delphi Method

Qualitative evaluation is not only a method of describing language form, but also a kind of philosophical thinking and logical analysis, which is used to reveal, analyze, and deal with the information characteristics of the evaluation object. Its purpose is to understand the essence of things and form an overall view of the evaluation object. Based on the observation and analysis of the performance, reality, state, or literature of the evaluation subject, the value orientation of the evaluation conclusion of the evaluation subject, such as scoring and writing Comments and system performance. Qualitative evaluation is a bid evaluation method that uses the knowledge, experience, and judgment of bid evaluation personnel to evaluate and compare the image of bid evaluation. Qualitative evaluation includes observation, analysis, induction, and description.

Delphi method, also known as expert investigation method, is a method to invite several experts to evaluate and judge a certain decision based on their own experience. In this method, several experts do not know that other experts are involved in the investigation [25]. This method is an anonymous program survey method, which is used to predict possible situations and factors and judge the importance of relevant influencing factors in the system. This paper will use this method to preliminarily set some factors, which may affect the quality of education and teaching.

#### 2.2.5. Method Comparison

Analytic hierarchy process is a method of calculating weight, and fuzzy comprehensive evaluation method is a method of comprehensive evaluation of problems. In fuzzy comprehensive evaluation, analytic hierarchy process (AHP) can be used to assign the weight of each factor. Therefore, the two are complementary. Compared with analytic hierarchy process and grey correlation analysis, analytic hierarchy process is too subjective. Sometimes the constructed matrix cannot pass the consistency test, and the grey correlation analysis method can make up for the defects brought by mathematical statistics and will not show the inconsistency between quantitative results and qualitative results.

### 2.3. Web-Based Assessment Program of College Physical Education Level

The advantage of big data lies not only in its massive data, but also in its ability to conduct professional analysis of the obtained data [26]. It is not only causality research, but also relationship research. For the evaluation of teaching quality in colleges and universities, the construction of an evaluation system based on big data is a necessary condition to realize the scientization, indexation, and informatization of teaching level evaluation [20]. This paper designs the function of the evaluation system. Due to the diversity of college education evaluation subjects and the complexity of teaching indicators, an evaluation model with hierarchical distributed structure is required. In addition to the data layer, it also needs a relational authority layer, a functional layer, and a display layer [27]. Model of this paper is based on Java language design implementation, and the main functions include evaluation system, data acquisition and screening, data service, and comprehensive analysis. And this system uses the browser/server structure and requires no additional installation applications, and the advantages of this method are convenient to get the data and will not increase the cost, because the number of users the disadvantage is that safety control ability may be insufficient, the specific system structure from left to right, as shown in Figure 2. In the next step, we will try to design the system as an application program, which can support Android system, IOS system, and Microsoft system to ensure wide usability.

There are five modules in the functional layer, which are teaching evaluation index management, teaching evaluation task management, basic management, teaching evaluation supervision data management, and the whole process of evaluation management. Teaching evaluation indicators are designed according to different evaluation identities, and the specific content will be reflected in the experiment; teaching evaluation task is regularly organized by the school to conduct teaching evaluation on curriculum and teacher teaching; the evaluation data are summarized in the data management module, and the correlation degree is analyzed [28].

## 3. Experiment and Analysis

### 3.1. Experimental Arrangement

#### 3.1.1. Experimental Subjects

In consideration of the rationality of sample selection, this paper does not choose science and engineering colleges or liberal arts colleges. Instead, take a comprehensive university in South China as an example, with all undergraduates and teachers of the school as the main survey objects. Based on the data obtained from the school's online teaching platform, data mining and analysis of the physical education quality evaluation process of the first grade of the school in 2021 are carried out. The school offers a total of 13 physical education courses (badminton, table tennis, basketball, football, yoga, Tai chi, taekwondo, roller skating, volleyball, aerobics, shot put, swimming, and javelin throw). The basic professional information of students and teachers is given in Table 1.

#### 3.1.2. Experimental Environment

The research in this paper is supported by big data technology and distributed processing architecture. The structure diagram of education and teaching evaluation system has been mentioned above. In this paper, the experimental computer system is Windows 7, the database uses MySQL5.7.17, Java as the design language, and Web as the main platform. The specific network structure is shown in Figure 3.

The system based on mobile terminal design USES B/S architecture, the user mobile terminal, can be achieved through the browser user login, evaluation process and the result query operation, maintenance work for system administrators to conduct the background, involving system data import and entry, and system function to maintain a complex operation. Implementation as a browser on a WEB server will still be supported. Based on this system, an AI big data teaching quality monitoring platform can be formed by integrating language processing, image recognition, machine learning, data mining, and other technologies, which can realize real-time monitoring and dynamic monitoring of teaching quality in colleges and universities.

### 3.2. Experimental Process

This experiment is roughly divided into the following parts: (1) Construction of index system. The evaluation index is the basis of teaching evaluation. Therefore, the first step of the experiment is to establish a scientific evaluation index system. The system mainly determines the possible influencing factors through expert investigation and then determines the weight and refines the index through quantitative methods. (2) System function design and model application. The design scheme is used in the teaching system, and the operation data of a semester are saved. (3) Summarize and analyze data. In teaching evaluation on account of massive information, data are the core, and the AI teaching quality monitoring system is designed to obtain the desired information and data for quality analysis.

#### 3.2.1. Index System Construction

In addition to the combination of education and science, the construction principle of the index system also needs the combination of qualitative analysis and quantitative analysis. It can not only reflect the characteristics of evaluation indicators, but also make decisions based on knowledge and experience. Therefore, an expert questionnaire was designed in this experiment, and the Delphi method was used to ask for expert opinions to determine the evaluation indicators.

*(1) Determination of First-Level Indicators and Weight Allocation.* Referring to the results of previous studies, this paper designs the first round of expert questionnaire for the setting of physical education teaching evaluation system in colleges and departments, forms the second round of questionnaire on this basis, and finally determines the secondary indicators. Based on the theoretical system of Delphi evaluation and the basic principles of education and teaching evaluation, the indicators of the first round of expert questionnaire are preliminarily determined as follows: teaching level, teaching attitude, teaching atmosphere, teaching effect, emotional stimulation, and facility environment. The scoring system is designed based on the importance of 9 scales in analytic hierarchy process, as shown in Table 2. Experts score the primary indicators through pairing and comparison.

Generally speaking, the number of experts is selected according to the size of the subject. Some studies have shown that if the number of experts is more than 9, its validity will reach the highest. The process of Delphi method generally includes: sorting, summarizing, and statistics after obtaining the opinions of experts on the problems to be predicted and then anonymous feedback to experts, soliciting opinions again, concentrating, and feedback again, until consensus is reached. In this paper, four experts who are interested in educational evaluation informational and have certain academic achievements were invited to score. Finally, four matrices were established according to the questionnaire survey results. In order to ensure the effectiveness of matrix results, consistency test was conducted on the four matrices. The final consistency ratio is 0.0398, 0.0653, 0.0952, and 0.0643, all less than 0.1, so the matrix can be used. Then, the analytic hierarchy process is used to get the weight of the six first-level indicators. Similarly, the consistency test is also carried out for the matrices in the analytic hierarchy process, and the final results are less than 0.05. These matrices are highly reliable. The results obtained based on the four matrices are shown in Figure 4.

After the feature vector corresponding to the largest feature root of the matrix is worked out and normalized, the weight distribution of the final level index is obtained as shown in Table 3. From this, we can see that the highest weight is index A (teaching level), followed by index *D* (teaching effect), and the smallest weight is index *F* (facilities and environment), indicating that the teaching level and effect are of high importance to the evaluation of education quality.

*(2) Determination of Secondary Indicators and Weight Allocation*. The second round of questionnaire was issued, and second-level indicators were formulated based on the determination of first-level indicators, with several second-level indicators corresponding to each first-level indicator. The secondary indicators developed are set out below.

Four indicators are set on teaching level A, which are as follows A1 (clear and accurate explanation of PE technical principles), A2 (scientific physical training load and time arrangement will not make students disgusted), A3 (able to master and share the latest sports education trends of the subject and stimulate students' interest), and A4 (teaching content is clear and targeted teaching).

The following indicators are set on teaching attitude B, respectively: B1 (teachers are energetic and passionate), B2 (pay attention to students' physical and mental state, can timely find students' problems, and provide guidance), B3 (pay attention to teaching feedback and make appropriate adjustments to the course content), and B4 (teaching process is organized and appealing).

Set the following indicators on teaching atmosphere C: C1 (teaching content is arranged to be interesting and attract students), C2 (focus on stimulating students' interest and flexibly using teaching methods), and C3 (students are active in learning and willing to actively cooperate with teaching). The following indicators are set on the teaching effect D: D1 (students can master the relevant theories and skills of physical education through learning), D2 (can enhance students' awareness of active exercise and form exercise habit), D3 (complete the teaching task set by the course); set the following indicators on emotional arousal E: E1 (harmonious teacher-student relationship), E2 (cultivation of students' cooperation and communication skills, and cultivation of students' emotions, attitudes, and values), E3 (love sports activities and understand relevant spirit through learning). The indicators set for facility environment F are as follows: F1 (relevant sports equipment and teaching AIDS are fully prepared), F2 (relevant sports venues meet the standards), and F3 (sports venues can be fully utilized).

The evaluation table of secondary indicators is shown in Table 4.

For the second round of questionnaire, 9-scale importance degree was also used to score and use the AHP to assign index weight. The results of the second-level matrix and weight distribution were obtained as shown in Figure 5.

Normalize the weight distribution of secondary indicators. The formula is as follows: w_i_ is the weight coefficient of secondary indicators under primary indicators, and *φ* is the weight coefficient of primary indicators.

(16) $$\begin{array}{c} W=w_{i}\cdot \varphi ,\;\left(i=1,2,\ldots ,20;j=1,2,\ldots \alpha \right). \end{array}$$

Thus, the weight of secondary indicators is shown in Figure 6.

As for the screening process of indicators, we combined expert opinions and consistency test of matrix. The consistency test values of primary indicators and secondary indicators were all less than 0.1, so the matrix could be judged to be effective. Meanwhile, experts did not put forward obvious opinions on indicators, but only modified the statement of indicators on the original basis. The degree of modification is not large. Compared with before and after, the specific expression of the secondary indicators of the latter is more scientific and standardized. Finally, the evaluation index system of physical education teaching quality in colleges and universities is sorted out as shown in Table 5.

### 3.3. Application and Data Analysis of Big Data Teaching Quality Evaluation Model

#### 3.3.1. AI Big Data Evaluation Process

After the evaluation index system is established and perfected, we design different electronic questionnaires for different PE courses for students to evaluate teaching and teachers to evaluate teaching. The evaluation data of this model come from different application subjects in the system, and each subject account is independent. They are evaluated according to the evaluation index system, classification, and system to collect the data and finally can be based on the comprehensive evaluation results of different appraisal main body, and the system is embedded within the grey relation analysis; on this basis to get feedback based on the fuzzy mathematics comprehensive evaluation, teachers' group and educational administration supervisor can query results, and on this basis to adjust course. The entire evaluation process account on AI monitoring is shown in Figure 7.

#### 3.3.2. Comparative Analysis of Model Application

In order to verify that the optimized comprehensive evaluation method is indeed better, experimental comparison is carried out in this paper, randomly selected two courses in the university, sorted out the data, and tested the methods before optimization and after optimization, respectively, from teaching level, teaching attitude, and teaching effect. The two groups of data randomly selected in this experiment are, respectively, the badminton and table tennis course data of the university. For this, multiple tests are conducted to collect monitoring stability error analysis data, and the sorting results are shown in Figure 8.

As can be seen from Figure 8, no matter which course, the teaching quality monitoring stability error of the experimental group is obviously lower than that of the control group, and the monitoring efficiency is better. In addition to comparing the error data, the accuracy of the model should also be tested and evaluated. In order to test the screening effect of the model on untrusted data, the experiment also collected experimental data to evaluate the average risk, as shown in Figure 9. The results suggest that the risk of teaching evaluation affects monitoring model designed in this experiment is about 1.93 lower than that of the control group; that is, the accuracy of the application model of this experiment is significantly higher, and the data with low reliability can be filtered from massive data, which can greatly promote the reliability of the evaluation system.

#### 3.3.3. Dynamic Analysis of Education Level Evaluation

Part of the education assessment data in the spring of 2021 and the education evaluation data in the autumn of 2021 were analyzed, and the evaluation results were tested by SPSS software. The results showed that the average evaluation results of PE teachers in the autumn of 2021 were higher than that in the spring of 2021, about 3.36 points higher. The teaching quality of PE courses in the first half of 2021 is high.

The overall data statistics of the two types of samples are found to conform to normal distribution, as shown in Figure 10. Smirnoff test was used to test the significance of the evaluation data in the samples. Final result data display that there was no significant difference between the two samples, indicating that the evaluation results of the evaluation index system were relatively stable. In this study, the effectiveness and reliability of the evaluation results of physical education quality were high.

## 4. Discussion

This paper is committed to the dynamic analysis of College Physical Education Quality Evaluation account on massive data, constructs a data depth mining model, and constructs a network evaluation system using java language, which provides a reliable informational of college physical education evaluation. In the process of implementing the evaluation model, the combination of qualitative evaluation and quantitative evaluation is used to establish an optimized teaching quality evaluation index system. The primary and secondary indicators are clearly screened by Delphi method, and the weights of hierarchical distribution indicators and secondary indicators are determined by analytic hierarchy process and fuzzy comprehensive evaluation method, so as to realize the scientific and informational of indicators.

In order to ensure the validity of data, various methods are used to verify the validity of data. The consistency of the matrix generated by AHP is tested, and the samples obtained in the experiment are *Z* tested. At the same time, the comparative experiment of the experimental evaluation model between the control group and the experimental group is carried out, and the physical education courses of two schools are selected for analysis. The experimental results show that the optimized evaluation model has small experimental error and high precision, and has good effect of filtering irrelevant information in the era of big data. The risk coefficient of the experimental group is low, and the risk coefficient of the control group is 1.93.

## 5. Conclusion

The experimental scheme was applied to the evaluation and analysis of the first-year physical education curriculum of a university in Southwest China, and the physical education teaching process of the University was continuously captured for one academic year. The results suggest that there is no significant difference between the two groups in the experiment. The above contents show that the physical education teaching evaluation scheme in this experiment has good stability, and the feedback information can effectively help teachers improve teaching quality. It can be clearly seen from the mean difference between the two samples in spring and autumn in 2021. The score in autumn is 80.02 and that in spring is 76.34.

## Figures and Tables

**Figure 1:** Data mining of massive data.

**Figure 2:** Web-based education quality evaluation system in colleges and universities.

**Figure 3:** Experimental environment and network structure diagram.

**Figure 4:** Weight of first-level evaluation indicator matrix.

**Figure 5:** Weights of second-level indicators in their respective groups.

**Figure 6:** Weight distribution of secondary indicators.

**Figure 7:** Educational evaluation process.

**Figure 8:** Teaching monitoring error chart.

**Figure 9:** Evaluation risk comparison.

**Figure 10:** Two-sample statistical chart.

**Table 1:** Experimental object.

Student information				
	Professional types	Male	Femininity	Sum

1	Finance	632	814	1446
2	Management	635	725	1360
3	Politics & Law	498	580	1078
4	Literature & History	336	625	961
5	Education	197	398	595
6	Science & Engineering	1056	645	1701
7	Medicine	143	112	255
8	Agronomy	381	300	681
	Sum	3878	4199	8077

Teacher information				
	PE course	Male	Femininity	Sum

1	Ping-Pong	8	6	14
2	Badminton	6	6	12
3	Basketball	8	5	13
4	Football	5	3	8
5	Volleyball	7	6	13
6	Shot put	5	1	6
7	Swimming	6	5	11
8	Javelin	2	3	5
9	Roller skating	4	2	6
10	Aerobics	1	4	5
11	Tai Chi	4	2	6
12	Taekwondo	5	3	8
13	Yoga	0	4	4
	Sum	61	50	111

**Table 2:** Level of importance.

Factor/factor (importance）	Quantized value
Equally	1
Slightly	3
More	5
Strongly	7
Extremely	9
Median	2, 4, 6, 8

**Table 3:** Weight distribution of first-level indicators.

Weight ratio						
Index	A	B	C	D	E	F
Weights	0.2754	0.1130	0.1578	0.2460	0.1100	0.0978

**Table 4:** Secondary index evaluation table.

A	Teaching level	A1 (sports technical essentials are explained clearly and accurately) A2 (sports training load and time arrangement are scientific and will not disgust students) A3 (be able to master and share the latest sports education trends of the taught discipline and stimulate students' interest) A4 (teaching content is difficult to point out and carry out targeted teaching)

B	Teaching attitude	B1 (teachers are full of energy and passion) B2 (pay attention to students' physical and mental state, find students' problems in time, and give guidance) B3 (pay attention to teaching feedback and adjust the course content appropriately) B4 (the teaching process is organized and appealing)

C	Teaching atmosphere	C1 (the arrangement of teaching content is interesting and attracts students) C2 (pay attention to the stimulation of students' interests and flexibly use teaching methods) C3 (students have high learning enthusiasm and are willing to actively cooperate with teaching)

D	Teaching effectiveness	D1 (students in learning master the relevant theoretical knowledge and skills of the physical education course) D2 (can enhance students' awareness of active exercise and develop sports habits) D3 (complete the teaching tasks set in the course);

E	Emotional stimulation	E1 (harmonious and interactive relationship between teachers and students) E2 (cultivate students' ability to cooperate with others and pay attention to the cultivation of students' emotions, attitudes, and values) E3 (students love sports activities and understand relevant spirit through learning)

F	Facility environment	F1 (relevant sports equipment and teaching aids are fully prepared) F2 (sports venues meet the standards) F3 (sports venues can be fully utilized)

**Table 5:** Evaluation form of physical education teaching quality in colleges and departments.

First-level indicator	Weights	Second-level indicator	Weights
Teaching level A	0.0257	A1	0.1069
		A2	0.0659
		A3	0.0391
		A4	0.0636

Teaching attitude B	0.1130	B1	0.0261
		B2	0.0309
		B3	0.0337
		B4	0.0223

Teaching atmosphere C	0.1578	C1	0.0568
		C2	0.0576
		C3	0.0434

Teaching achievement D	0.2460	D1	0.0813
		D2	0.0896
		D3	0.0752

Emotional stimulation E	0.1100	E1	0.0401
		E2	0.0419
		E3	0.028

Facility environment F	0.0978	F1	0.0363
		F2	0.0341
		F3	0.0272
Sum	1		1

## Data Availability

No data were used to support this study.
